RETRACTED

# Efficacy and Side Effects of Irinotecan Combined with Nedaplatin versus Paclitaxel Combined with Cisplatin in Neoadjuvant Chemotherapy for Locally Advanced Cervical Cancer and Tumor Marker Analysis: Based on a Retrospective Analysis

**DOI:** 10.1155/2022/5936773

**Published:** 2022-06-01

**Authors:** Yu Jiang, Baozhi Song, Zhiqin Chen

**Affiliations:** Provincial Clinical College of Fujian Medical University (Department of Gynecology, Fujian Provincial Hospital), Fuzhou, 350001 Fujian, China

## Abstract

**Objective:**

A case-control study was adopted to investigate the efficacy and side effects of irinotecan combined with nedaplatin (NP) versus paclitaxel combined with cisplatin for locally advanced cervical cancer (CC) neoadjuvant chemotherapy (NACT) and to analyze the changes in tumor marker levels.

**Methods:**

A total of 96 patients with locally advanced CC who were treated from October 2019 to October 2021 were enrolled in our hospital as the research subjects, and their clinical data were collected for retrospective analysis and grouped according to their treatment regimens. Among them, 53 patients received paclitaxel combined with cisplatin as the control group, and the other 43 patients received irinotecan combined with NP as the observation group. The clinical effectiveness of neoadjuvant chemotherapy and alterations in tumor markers (CEA, AFP, CA125, and SCCA) were compared between the two groups. The incidence of common chemotherapy side effects was observed and compared between the two groups, including nausea and vomiting, abdominal pain and diarrhea, liver function impairment, bone marrow suppression, transient hyperglycemia, rash, ECG abnormalities, peripheral neurotoxicity, and muscle aches and pains.

**Results:**

The clinical efficiency of neoadjuvant chemotherapy was 97.67% in the observation group and 81.13% in the control group, with no statistically significant difference between the groups (*P* > 0.05). There was no significant difference in CEA, AFP, and CA125 between the two groups before and after chemotherapy, but the decrease of SCCA before and after chemotherapy was statistically significant. There was no significant difference in the incidence of liver function damage, myelosuppression, abnormal ECG, and rash between the two groups (*P* > 0.05). There are statistically significant differences in the incidence of nausea and vomiting, transient hyperglycemia, peripheral neurotoxicity, and muscle aches between the observation and control groups (*P* < 0.05). The incidence of nausea and vomiting, transient hyperglycemia, peripheral neurotoxicity, and muscle aches was higher in the control group than in the observation group, with statistically significant differences (*P* < 0.05). The difference in the incidence of diarrhea and abdominal pain between the observation group and the control group was statistically significant (*P* < 0.05), and the incidence of diarrhea and abdominal pain in the observation group was higher than that in the control group.

RETRACTED

**Conclusion:**

Irinotecan in combination with nedaplatin can be an effective neoadjuvant chemotherapy regimen for advanced localized cervical cancer, particularly in patients with combined diabetes.

## 1. Introduction

Cervical cancer (CC) is an obvious type of cancer in the female reproductive system. It ranks first in the incidence of malignant tumors of the female reproductive system and ranks second in all malignant tumors in women [1]. Statistics show that the number of new CC patients in my country is about 131,500 each year, and in recent years, the incidence of the disease has indicated an increasingly younger trend, and locally advanced CC is a common type [2]. When such patients are treated with surgery alone, the long-term survival rate of patients is less than 40% [3].

In the traditional treatment mode, chemotherapy is usually adopted as palliative treatment or supplementary adjuvant treatment after surgery for CC patients [4]. The concept of neoadjuvant chemotherapy (NACT) first appeared in 1982, which was put forward by Frey in the United States, which refers to the treatment of malignant tumors by systemic intravenous chemotherapy or local transarterial interventional chemotherapy before the main treatment of malignant tumors such as radiotherapy or local operation [5]. NACT is a new chemotherapy method, which is a systemic treatment measure carried out before radiotherapy or surgery, and its clinical application has been increasing in recent years. The purpose of NACT is to shrink the tumor as much as possible, reduce the scope of tumor invasion, then create surgical opportunities for patients with malignant tumors who could not be treated by surgery, and reduce the risk of parametrial tissue involvement and lymph node metastasis [6]. This promotes the improvement of the curative effect of patients. It can be said that NACT is an important adjuvant therapy. In recent years, with the continuous application of effective chemotherapeutic drugs (such as platinum and paclitaxel) in clinical practice, and the gradual improvement of drug routes and methods, NACT regimens are often used in the treatment of CC patients at this stage [7]. For patients with locally advanced CC, the NACT regimen is very complicated, and some chemotherapy regimens are not effective, or can cause serious toxic and side effects, making it difficult for patients to tolerate.

RETRACTED

In recent years, the application value of NACT has been gradually recognized at home and abroad [8]. A large number of studies and clinical trials have been carried out on NACT in China, and it has been found that compared with simple surgery, NACT followed by surgery can promote tumor shrinkage and enhance the resection rate of lesions by surgery [9]. It can reduce the infiltration of CC to the parametrium and double appendages, reduce the risk of tumor thrombus formation in the blood vessels, reduce the recurrence rate of postoperative stumps, and help enhance the survival rate and quality of life of patients [10]. The study by Xuesong and Yajuan found that, compared with patients without NACT, after NACT, arterial intervention, for patients with locally advanced CC, the surgical resection rate was 48% to 100% [11]. This will lead to an increased risk of postoperative complications. About 9%/18% of the patients were evaluated as complete remission by postoperative pathological examination, and the rate of lymph node metastasis decreased significantly.

At present, there are many drugs available for NACT in patients with locally advanced CC, and the chemotherapy regimen is mainly platinum plus paclitaxel [12]. The TP regimen was paclitaxel plus cisplatin, and the TC regimen was paclitaxel plus carboplatin. Paclitaxel is a natural plant product. It was first extracted from the bark of the yew tree in 1963. The drug is the most effective drug among the natural anticancer drugs discovered in recent years. Paclitaxel can promote the aggregation and coagulation of cellular tubulin into bundles and can prevent depolymerization [12]. When acting on tumor cells, paclitaxel can specifically play a role in the G2 phase and M phase of the cell cycle, preventing microtubules from forming spindles and spindle filaments in mitosis, and blocking the process of tumor cell division and proliferation. At the same time, paclitaxel can have an effect on macrophages, resulting in the release of tumor necrosis factor, interferon-*α*, interferon-*β*, and other factors, thus inhibiting or killing tumor cells. In the treatment of patients with CC and endometrial carcinoma, 50 patients were randomly assigned by drawing lots [13]. The control group was treated with azithromycin, and the observation group was treated with paclitaxel. After comparison, the total effective rate of the observation group was remarkably higher compared to the control group, and the mortality rate and recurrence rate were remarkably lower compared to control group, while the incidence of adverse reactions in the observation group was remarkably lower compared to the control group. Through this study, the authors propose that paclitaxel can enhance the therapeutic effect of CC and improve the prognosis of patients.

RETRACTED

In order to maximize the therapeutic effect, clinicians usually combine paclitaxel and platinum drugs to exert a synergistic effect [14]. After cisplatin NACT, surgery was performed. Cisplatin is a first-generation platinum-based antitumor drug and is currently adopted in NACT for most tumors. Through clinical practice, we have found that platinum drugs can cause certain renal toxicity, because platinum can be deposited in the kidneys, causing kidney damage. The degree of nephrotoxicity of platinum drugs is closely related to the type of drug. Cisplatin is the most obvious drug of nephrotoxicity, and drug dose and cumulative renal insufficiency are the most important causes of nephrotoxicity. At present, hydration therapy is adopted to prevent nephrotoxicity in clinical practice, but the risk of renal injury is still about 1/3. Therefore, finding new and effective chemotherapy drugs has become the focus of current clinical work. NP, irinotecan, and paclitaxel are the most commonly used drugs in the treatment of advanced CC under current conditions. NP belongs to a new type of platinum drug under investigation and has a strong antitumor effect [15]. Our hospital has achieved good results in the application of irinotecan combined with NP as the first choice for the treatment of locally advanced CC. The report is as follows.

## 2. Patients and Methods

### 2.1. Normal Information

A total of 96 patients with locally advanced CC who were treated in our hospital from October 2019 to October 2021 were enrolled as the research subjects, and their clinical data were collected for retrospective analysis and grouped according to their treatment regimens. Among them, 53 patients received paclitaxel combined with cisplatin as the control group, and the other 43 patients received irinotecan combined with NP as the observation group. In the observation group, the age ranged from 32 to 73 years, with an average of (55.13 ± 1.21) years. In the control group, the age ranged from 31 to 75 years, with an average of (55.36 ± 1.37) years. The general data of patients were not statistically significant and were comparable, as indicated in Table 1 for details. This study was permitted by the medical ethics committee of our hospital, and all patients noticed informed consent.

Selection criteria were as follows: (1) diagnosed as locally advanced CC by MRI, CT and other imaging examinations and combined with pathological sections and clinical diagnosis; (2) without cognitive, language, and intellectual impairment and with basic reading and writing ability; (3) FIGO stage I B3 ~ II A2; (4) no other chemotherapeutic drugs were used within 1 week before inclusion; (5) the clinical data were complete; and (6) there were no abnormalities in blood routine, ECG, and other biochemical tests before treatment.

RETRACTED

Exclusion criteria were as follows: (1) complicated with other malignant diseases such as liver cancer and gastric cancer; (2) dysfunction of important organ such as the kidney; (3) refusing to participate; (4) excluding mental disorders, Alzheimer's disease, or other cognitive impairment; (5) excluding female patients during pregnancy and lactation; and (6) the expected survival time is less than 3 months.

### 2.2. Treatment Methods

The control group was as follows: paclitaxel (manufacturer: Hospira Australia Pty Ltd., approved by Chinese medicine H20090175, specification: 30 mg) combined with cisplatin (manufacturer: Qilu Pharmaceutical Co., Ltd., permitted by Chinese medicine: H37021362, specification: 20 mg). Use 500 mL 0.9% sodium chloride injection plus 135~175 mg/m^2^ paclitaxel, 500 mL 0.9% sodium chloride injection plus 70 mg/m^2^ cisplatin for intravenous drip, and 20 mg dexamethasone orally 12 h and 6 h before chemotherapy. Before 30 minutes of chemotherapy, take 50 mg of diphenhydramine orally (manufacturer: Linfen Baozhu Pharmaceutical Co., Ltd., Chinese medicine approved word: H1402149, specification: 25 mg) and intravenously 400 mg of Losec (manufacturer: AstraZeneca Pharmaceutical Co., Ltd. Chinese medicine quasiword: H20033394, specification: 0.2 g). During the treatment process, vital signs such as heart rate, blood pressure, and pulse should be monitored every 15 minutes for at least 3 hours. And more than 3000 mL of fluid needs to be rehydrated every day for 3 days. Combination chemotherapy requires 2 courses, and each course needs to be separated by 21 days.

The observation group was as follows: on the day of chemotherapy, irinotecan (Jiangsu Hengrui Pharmaceutical Co., Ltd., approved by H20040711) 160 mg m^−2^ intravenously, NP (Nanjing Xiansheng Dongyuan Pharmaceutical Co., Ltd., approved by H20030884) 80 mg m^−2^ intravenous infusion, and intramuscular injection of anisodamine (Tianjin Jinyao Amino Acid Co., Ltd., H12020889) half an hour before irinotecan chemotherapy, repeated chemotherapy on 21 d, and a total of 2 courses of treatment.

### 2.3. Observation Indicator

#### 2.3.1. Efficacy Evaluation Criteria

Using the evaluation criteria for solid tumors [16]: (Response Evaluation Criteria in Solid Tumors, RECIST) 1.1 as an evaluation criterion (complete response, CR), (partial response, PR), (stable disease, SD), and (progressive disease, PD), CR indicates that all lesions disappeared, and no new lesions were found; PR was as follows: compared with the baseline period, the sum of the relative values of the maximum diameter of the tumor decreased by ≥30%; SD was as follows: between PR and PD; PD was as follows: compared with the baseline period, the tumor diameter increased by >20% compared with the maximum and minimum, or new lesions appeared. Objective response rate (ORR) was as follows: ORR = (CR + PR)/total number of people∗100%. Disease control rate (DCR) was as follows: DCR = (CR + PR + SD)/total population∗100%. All patients completed baseline MRI examination after entering the group, and the same imaging examination was performed again at the end of treatment. The same researcher completed the tumor assessment at baseline and during treatment.

RETRACTED

#### 2.3.2. Tumor Marker Levels

Before treatment and after 2 course of treatment, 5 mL venous blood was drawn from both groups of patients on an empty stomach, a vacuum blood collection tube was placed, centrifuged at 4000 r/min for 10 min at room temperature, and the upper serum was collected for the detection of AFP, CEA, SCCA, and CA125 in serum.

#### 2.3.3. Adverse Reactions

The incidence of common chemotherapy adverse reactions such as gastrointestinal reactions (vomiting, diarrhea), liver function damage, bone marrow suppression, abnormal electrocardiogram, transient hyperglycemia, skin rash, peripheral neurotoxicity, and muscle pain was observed. Here is the following formula: incidence of adverse reactions = (number of adverse reactions/total number of people)∗100%.

### 2.4. Statistical Analysis

SPSS 22.0 statistical software was adopted for data processing and chart drawing; measurement data were presented as mean ± standard deviation (*x* − ±*s*), and *t*-test was adopted for comparison between groups; enumeration data were presented as number of cases and rate (%), and between groups, the chi-square test was employed for comparison, and *P* < 0.05 was considered as statistically significant.

## 3. Results

### 3.1. Comparison of Baseline Data between the Two Groups

First, we compared the baseline data of patients. There was no significant difference in age, body mass index (BMI), HPV infection rate, pathological type, FLGO stage, differentiation degree, and menopause (*P* > 0.05). The specific results are indicated in Table 1.

### 3.2. Comparison of Therapeutic Effects between the Two Groups

We compared the therapeutic effects. The observation group had 6 cases of CR, 28 cases of PR, 8 cases of SD, and 1 case of PD, with a total remission rate of 97.67%; the control group had 3 cases of CR, 22 cases of PR, 18 cases of SD, and 10 cases of PD, and the total response rate was 97.67%. The remission rate was 81.13%. The total remission rate in the observation group was higher than that in the control group (*P* < 0.05). All results are indicated in Figure 1.

RETRACTED

### 3.3. Comparison of Tumor Markers between the Two Groups

We compared the levels of tumor markers, and there exhibited no significant difference in serum AFP, CEA, and CA199 levels before treatment (*P* > 0.05). The levels of AFP, CEA, and CA199 after treatment were lower than those before treatment. Compared with the two groups, the improvement of the observation group was significantly better than that of the control group. All the results are indicated in Table 2.

### 3.4. Comparison of the Incidence of Adverse Reactions

We compared the incidence of adverse reactions. After receiving ≥2 cycle of chemotherapy, all patients were evaluated for safety by the same group of investigators. Both groups experienced different degrees of toxic and side effects during treatment. The above adverse reactions were alleviated after symptomatic treatment, and no patient discontinued treatment due to chemotherapy intolerance. Three patients in the observation group needed to reduce the dosage during the study period, and 11 patients in the control group needed to adjust the dosage according to the situation. There was no significant difference in the incidence of vomiting, liver function damage, myelosuppression, abnormal ECG, and rash (*P* > 0.05). The incidence of diarrhea in the observation group and control group was 18.60% and 3.77%, respectively (*P* < 0.05), and the incidence of diarrhea in the observation group was higher compared to the control group; the incidences of transient hyperglycemia, peripheral neurotoxicity, and muscle soreness in the observation group and the control group were 16.28% and 52.83%, 13.95% and 1.89%, and 11.63% and 20.75%, respectively (*P* < 0.05). All results are indicated in Figure 2.

## 4. Discussion

In recent years, the incidence of CC has been high worldwide [16]. About 600000 women are diagnosed with CC each year, with a mortality rate of 34 percent. 90% of patients are concentrated in developing countries where health standards are underdeveloped [17]. Its pathogenesis is closely related to HPV infection. Due to the weak awareness of health screening and the shortage of HPV vaccine resources, the number of newly diagnosed cases in my country is increasing year by year. The International Federation of Obstetrics and Gynecology (FIGO 2018 standard) defines stage IB3 and IIA2 CC, that is, CC with a tumor diameter greater than 4 cm, as locally advanced CC because of its large mass, high lymph node metastasis rate, rapid progression, and easy recurrence; usually, patients have poorer quality of life and shorter survival time. At present, the preferred treatment for early CC is surgery, while the dominant treatment options for locally advanced CC in different countries and regions are still quite different, which is the focus of current debate. The National Comprehensive Cancer Network (NCCN) believes that patients with locally advanced CC should choose concurrent radiotherapy and chemotherapy as the first choice for treatment, but radiotherapy will also cause unavoidable irreversible damage to normal cells and tissues in the human body, such as radiation cystitis, enteritis, skin damage, and permanent damage to the ovary, vagina, and other reproductive systems, and psychological disorders caused by long-term gastrointestinal function, urinary function, and sexual dysfunction of patients should also be paid attention to clinically [18]. In addition, the current uneven level of global radiotherapy equipment and technology, as well as the relative backwardness of research on precision radiotherapy in developing countries, the application of radiotherapy is relatively limited. Therefore, the treatment mode of neoadjuvant chemotherapy (NACT) combined with radical surgery (RS) has been gradually introduced into clinical practice in most developing countries.

RETRACTED

NACT makes tumor cells hypoxic and necrotic through local or systemic medication, and the tumor volume is remarkably reduced, which not only increases the opportunity for surgery for young patients but also greatly reduces the difficulty of surgery and the possibility of distant tumor metastasis [19]. In addition, NACT reduces the number of hypoxic cells and increases tumor sensitivity to radiotherapy. Several clinical studies have indicated that platinum-based chemotherapy can effectively enhance the survival of LACC patients and reduce short-term and long-term recurrence. Given the remarkable short-term efficacy of NACT, its use in developing countries is becoming more widespread, especially in younger patients [20]. Clinical big data research indicates that the application rate of NACT in my country has been increasing year by year since 2004 and has always remained at a high level. However, whether NACT can promote the long-term survival and prognosis of LACC patients is still controversial [21]. Some studies believe that preoperative application of chemotherapeutic drugs can reduce the risk of distant metastasis of cancer cells and the infiltration rate of parametrial tissue and lymphatic vessels but does not promote the overall survival rate of patients [22]. The results of current clinical studies vary. In this study, retrospective analysis was adopted to analyze the data of patients with locally advanced CC and to explore NACT by comparing the efficacy of irinotecan combined with NP and paclitaxel combined with cisplatin in patients with locally advanced CC. Analyze the curative effect and side effect of the patients and the level of tumor markers of the patients and provide a more reliable clinical basis for choosing a more reasonable treatment plan.

RETRACTED

The introduction of the concept of NACT in 1982 opened up a new mode of treatment for LACC, especially in regions with limited radiotherapy technology such as Asia, Europe, and Latin America [23]. The application of NACT makes tumor cells hypoxic and necrotic, effectively reducing tumor volume and preventing the formation of distant micro metastases. Chang et al. randomly assigned 124 LACC patients into the NACT+RS group and CCRT group [24]. The results indicated that the 5-year survival rates were 70% and 61%, respectively. A meta-analysis by Marchetti also concluded that the two treatment modalities had similar benefits [25]. Rasoulian et al. assigned 476 patients with LACC into PRS group, group NACT+RS, and group CCRT, the study indicated that the 5-year OS and PFS of the three groups of patients were (64.37%, 88.67%, 80.21%, *P* < 0.0001) (52.94%, 85.0%, 77.44%, *P* < 0.0001), and it is concluded that NACT can remarkably enhance the overall survival time and tumor-free survival time of patients among the three treatments [26]. The research and application of NACT have a history of more than 20 years. Its good short-term effect is obvious to all. It can effectively reduce the occurrence of high-risk pathology, but can it improve the long-term survival rate and quality of patients? There is no unified consensus on the life of patients. This is still the focus of controversy.

Clinical big data studies show that the application rate of preoperative NACT in my country has increased linearly since 2004 and has remained at a high level since then [27]. A retrospective study by Wang et al. indicated that compared with direct surgery, preoperative NACT remarkably reduced the rate of lymph vascular space involvement (*P* = 0.021) and the rate of deep myometrial invasion (*P* = 0.034). The incidence of high-risk factors such as parametrial invasion, lymph node metastasis, and positive vaginal margins were also reduced, but there was no statistical basis [28]. A meta-analysis indicated that in 21 randomized controlled trials, most studies believed that NACT combined with RS can remarkably improve the overall survival rate of patients with stage IB2 to IIB LACC, but a large number of clinical data are still needed to be further confirmed [29]. Qin et al. randomly assigned 65 LACC patients into two groups: NACT combined with surgery and direct surgery [30]. The results indicated that NACT can remarkably prolong the disease-free survival of patients. Although the overall survival of patients is prolonged, there is no statistical basis. A phase III clinical trial of the Japanese Clinical Oncology Group found that compared with the direct surgery group, the proportion of patients receiving adjuvant radiotherapy after the NACT combination therapy was remarkably lower (58% vs. 80%) but still unable to high-risk pathological factors such as pelvic lymph node metastasis and deep stromal infiltration were excluded [31].

RETRACTED

In clinical practice, platinum-based chemotherapy is the first choice for LACC patients, and it is often adopted in combination with paclitaxel, bleomycin, vincristine, and irinotecan [32]. Studies have found that cisplatin-based chemotherapy can produce serious adverse events in LACC patients. A retrospective study in 2012 compared 252 patients with LACC who received paclitaxel combined with NP and cisplatin (TP) regimens, and the results indicated that the incidence of toxic reactions of NP and TP was 32.69% and 85.14%, respectively (*P* < 0.0001). The DFS of patients receiving NP and TP regimen was 81.41% and 67.28%, respectively (*P* = 0.014); OS of patients receiving NP and TP regimen was 93.89% and 81.54%, respectively (*P* = 0.0084). Compared with TP chemotherapy plus radical hysterectomy, NP chemotherapy plus radical hysterectomy provides higher remission rates, incidence of toxicity, and better long-term DFS and OS in LACC patients [33]. However, the current number of clinical studies is small, which needs to be proved by further research. Ferrandina et al. suggested that dose-intensive NACT can achieve a better pathological response rate without increasing the toxicity of patients [34].

With the further deeper of research, it is found that although there are many chemotherapy drugs, there are few chemotherapy drugs that can effectively enhance the short-term efficacy and long-term survival rate of patients. Therefore, the selection of effective chemotherapy drug combination has become the focus of current clinical research. NP, irinotecan, and paclitaxel are the most commonly used drugs in the treatment of advanced CC under current conditions. NP belongs to a new type of platinum drug under investigation and has strong antitumor effect. The pharmacological action of NP is basically the same as that of DDP, and it can interact with nucleosides in vivo and combine to form nucleoside-platinum conjugates. NP can bind to DNA in tumor cells and effectively block the replication of intracellular DNA, thereby achieving the effect of killing tumor cells. The solubility of NP is remarkably better compared to DDP, more than 10 times, and it can be adopted together with cisplatin and carboplatin without crossresistance; so, its clinical application is also increasing. In addition, NP is remarkably more effective than DDP in the treatment of CC, ovarian cancer, and endometrial cancer. Irinotecan is a DNA topoisomerase I inhibitor that can bind to topo-DNA complexes in tumor cells. The combined complex can produce a variety of ionic substances, and these ionic substances can be further combined with the DNA in the cell to stabilize the complex. In addition, irinotecan can also block the synthesis and replication of cancer cell DNA, thereby killing tumor cells. The purpose of this study was to observe the clinical efficacy of different chemotherapy schemes. The results of this study show that the total effective rate of the observation group is significantly higher than that of the control group, indicating that irinotecan combined with NPNACT can improve the clinical efficacy of patients with locally advanced CC.

RETRACTED

SCCA was first isolated from cervical squamous carcinoma tissue in 1977 and belongs to the family of serine protein inhibitors. SCCA inhibits apoptosis and participates in the differentiation of the columnar epithelial layer in normal squamous epithelial cells, and in tumor cells, it participates in the growth of tumors and has a diagnostic sensitivity of 50-70% for primary squamous cervical carcinoma. Serum SCCA concentration in patients with cervical cancer is positively correlated with clinical stage, and the rise and fall of SCCA level correspond to disease progression or improvement. Dynamic monitoring of serum SCCA levels can be used as an indicator for monitoring the condition of cervical cancer. Before and after treatment, although there was no significant change in the levels of AFP, CEA, and CA125 in the observation and control groups, there was a significant decrease in the levels of SCCA in both groups (*P* < 0.05), and the decrease in the test group was more significant than that in the observation group (*P* < 0.05). It indicates that NACT inhibited the growth activity of cervical cancer cells and created good conditions for further treatment (surgery or chemotherapy) subsequently, and the improvement effect of irinotecan combined with NP was better than that of paclitaxel combined with cisplatin. In terms of side effects, the incidence of diarrhea with irinotecan was higher compared to the paclitaxel group, but the incidence of diarrhea was remarkably reduced after the author applied amidoamine 0.5 h before chemotherapy. For patients with delayed diarrhea, antidiarrheal drugs can be adopted, and attention should be paid to the balance of water and electrolyte intestinal flora. Paclitaxel has allergic reactions and side effects. Dexamethasone must be used before to prevent allergic reactions. However, in clinical practice, the author found that in patients with locally advanced CC combined with diabetes, the application of dexamethasone led to a significant increase in blood sugar. Therefore, patients with diabetes should be cautious and avoid high-dose long-term application of dexamethasone. The same idea can be found in the study put forward by Zhao et al. [35]. They have applied new methods in the study, and the conclusions drawn can also give some support to this study.

RETRACTED

Conclusively, irinotecan combined with NPNACT can improve the curative effect, restore immune function, and promote clinical prognosis in patients with locally advanced CC without increasing adverse reactions. It can be used as one of the effective choices for locally advanced CC, especially for NACT in patients with diabetes. It is worthy of clinical promotion.

## Figures and Tables

**Figure 1:** Comparison of treatment effects between the two groups The observation group had 6 cases of CR, 28 cases of PR, 8 cases of SD, and 1 case of PD, with a total remission rate of 97.67%; the control group had 3 cases of CR, 22 cases of PR, 18 cases of SD, and 10 cases of PD, and the total response rate was 97.67%. The remission rate was 81.13%.

**Figure 2:** Comparison of the incidence of adverse reactions between the two groups. The incidence of diarrhea in the observation group and control group was 18.60% and 3.77%, respectively, and the incidence of diarrhea in the observation group was higher compared to the control group; the incidences of transient hyperglycemia, peripheral neurotoxicity, and muscle soreness in the observation group and the control group were 16.28% and 52.83%, 13.95% and 1.89%, and 11.63% and 20.75%, respectively.

**Table 1:** Comparison of baseline data between the two groups.

Relevant factors	O group (*n* = 43)	C group (*n* = 53)	*t/χ*2	*P*
Average age (years)	54.18 ± 8.61	54.73 ± 9.03	0.303	>0.05
BMI	22.72 ± 0.45	22.56 ± 0.52	0.115	>0.05
Pathological typing			0.487	>0.05
Squamous cell carcinoma	35 (81.40)	40 (75.47)		
Adenocarcinoma	8 (18.60)	13 (24.53)		
FLGO staging			0.583	>0.05
I B3 period	19 (44.19)	26 (49.06)		
II A period	24 (55.81)	27 (50.95)		
HPV infection rate	21 (48.83)	20 (37.73)	1.195	>0.05
Degree of differentiation			1.917	>0.05
Low differentiation	22 (51.16)	20 (37.74)		
Middle differentiation	12 (27.91)	21 (39.62)		
Highly differentiated	9 (20.93)	11 (20.75)		
Menopause			0.527	>0.05
Yes	27 (62.79)	37 (69.81)		
No	16 (37.21)	16 (30.19)		

RETRACTED

**Table 2:** Comparison of tumor marker levels before and after treatment in the two groups of patients ($\bar{x}\pm s$).

Group	*N*	AFP (ng/mL)		CEA (ng/mL)		CA125 (U/mL)		SCCA (ng/ml)	
		BT	AT	BT	AT	BT	AT	BT	AT
O group	43	4.08 ± 1.45	3.93 ± 1.24	2.96 ± 0.15	2.88 ± 0.35	16.54 ± 10.58	16.74 ± 9.28	3.56 ± 2.14	2.13 ± 1.12^a^
C group	53	4.18 ± 1.03	4.21 ± 1.87	2.58 ± 0.93	2.77 ± 0.71	15.67 ± 9.13	16.84 ± 7.46	3.68 ± 2.46	1.23 ± 1.05^b^
*t*		0.125	0.292	0.927	0.786	0.150	0.203	0.252	4.053
*P*		>0.05	>0.05	>0.05	>0.05	>0.05	>0.05	>0.05	<0.01

Note: comparison of the observation group before and after treatment, ^a^*P* < 0.05; comparison before and after treatment in the control group, ^b^*P* < 0.05. The levels of tumor markers were as follows, and there exhibited no significant difference in serum AFP, CEA, and CA199 levels before treatment (*P* > 0.05). The levels of AFP, CEA, and CA199 after treatment were lower than those before treatment. Compared with the two groups, the improvement of the observation group was significantly better than that of the control group.

## Data Availability

No data were used to support this study.
